The article "Exercise Intervention Improves Blood Glucose Levels and Adverse Pregnancy Outcomes in GDM Patients: A Meta-Analysis" was published in 2022. Journal: Comput Math Methods Med.

# Exercise Intervention Improves Blood Glucose Levels and Adverse Pregnancy Outcomes in GDM Patients: A Meta-Analysis

**DOI:** 10.1155/2022/9287737

**Published:** 2022-09-22

**Authors:** Xiaoyan Li, Rong Luo, Binbin Qiao, Haiwei Ou

**Affiliations:** ^1^Department of Endocrine, The First Affiliated Hospital of Hainan Medical University, Haikou 570102, China; ^2^Department of Gynaecology and Obstetrics, Haikou Maternal and Child Health Hospital, Haikou 570203, China; ^3^Department of Obstetrics, Danzhou People's Hospital, Danzhou 571700, China

## Abstract

**Objective:**

The objective of this study is to systematically evaluate the effect of exercise on gestational diabetes (GDM).

**Methods:**

The databases of PubMed, Cochrane Library, Web of Science, Embase, CNKI, VIP, and Wanfang were searched to collect publications regarding physical exercises and GDM. The two researchers screened the literature, extracted the data, and analyzed the risk of bias of the included data using RevMan 5.3 software. The primary outcomes analyzed included the fasting blood glucose, 2-h postprandial blood glucose, glycosylated hemoglobin, premature delivery, cesarean section, neonatal macrosomia, premature rupture of membranes, and neonatal hypoglycemia.

**Results:**

A total of 9 studies with 1289 GDM patients were included. Compared with the control group, exercise could significantly reduce the 2-h postprandial blood glucose (MD = −0.62, *95% CI* (-0.91 to -0.34), *Z* = 4.29, *P* < 0.0001), improve HbA1c(RR = −0.47, *95% CI* (-0.81 to -0.13), *Z* = 2.69, *P* = 0.007), reduce the cesarean section rate (RR = 0.83, *95% CI* (0.71-0.98), *Z* = 2.25, *P* = 0.02), and decrease the incidence of neonatal macrosomia in GDM patients (RR = 0.57, 9*5% CI* (0.34-0.95), *Z* = 2.17, *P* = 0.03).

**Conclusion:**

Exercise intervention can improve the blood glucose level of GDM patients, such as 2-h postprandial blood glucose and HbA1c. Meanwhile, exercise can also reduce adverse pregnancy outcomes, such as premature birth and macrosomia. Therefore, prescribing exercise to GDM patients can effectively manage GDM and improve adverse pregnancy outcomes.

## 1. Introduction

Gestational diabetes (GDM), defined as any degree of glucose tolerance, is one of the most common conditions during pregnancy [1, 2] that increase the risk of adverse perinatal outcomes for both the mothers and infants, such as premature birth, macrosomia, and premature rupture of membranes. [3, 4]. The global prevalence of GDM is 2-32%, and about 18.4 million live births are affected by GDM in China [5]. Recently, the incidence of GDM in China has also been gradually increasing [3, 6]. Not only patients with GDM have an increased probability of developing type 2 diabetes in the future, their children are also more prone to develop metabolic diseases such as diabetes, obesity, and hypertension [7]. Therefore, blood glucose control for pregnant women is essential to protect the health and safety of mothers and fetuses. When pregnant women were diagnosed with GDM, they are frequently recommended to do more exercise and eat regularly [8]. Drug intervention may only be considered when the target blood glucose level can still not be reached after exercise intervention. Nonetheless, the use of medications is curtailed by concerns of adverse effects on the mother and fetus [9]. Therefore, effective interventions and safe guidance to control blood glucose level of pregnant women are desirable.

The article "Exercise Intervention Improves Blood Glucose Levels and Adverse Pregnancy Outcomes in GDM Patients: A Meta-Analysis" was published in 2022. Journal: Comput Math Methods Med.

Physical exercise is considered to be an important part of GDM lifestyle intervention. Previous studies have shown that physical activities before or during pregnancy can reduce the risk of GDM [10]. Furthermore, a regular exercise during pregnancy can also reduce the blood glucose level of pregnant women [11]. A previous study reported that healthy pregnant women should perform a moderate-intensity exercise at least 4 times a week, at least 30 minutes each time [7]. Regrettably, only a limited proportion of pregnant women can achieve this exercise frequency or intensity. Thus, in this study, we systematically analyzed the effect of physical exercise on the blood glucose level of GDM patients and adverse pregnancy outcomes, thus providing reference for guiding the prescription of physical exercise for GDM patients.

## 2. Research Objects and Research Methods

### 2.1. Literature Search

We searched the Chinese and English electronic databases CNKI, VIP, Wanfang, PubMed, Cochrane Library, Web of Science, and EMBASE databases from inception to July 5, 2022, using a combination of search words that included (sports OR exercise OR activity OR training OR physical) AND (gestational diabetes mellitus OR GDM).

### 2.2. Inclusion and Exclusion Criteria

Inclusion criteria are as follows: (1) The research object was diagnosed with GDM; (2) a complete exercise intervention program that included exercise time, frequency, and intensity was performed; (3) outcome index ≥3; and (4) the type of study was randomized controlled trial (RCT). Exclusion criteria are as follows: (1) patients with conditions other than GDM; (2) incomplete outcome indicators or data that were unable to extract; (3) medications were added to the intervention, in addition to physical exercise; and (4) the full text of the literature cannot be obtained.

### 2.3. Quality Evaluation and Risk of Bias Assessment

A total of 9 RCT literature were included in this study, of which four had only one missing or unclear outcome index [3, 11–13], and five had two missing or unclear outcome indexes [2, 4, 8, 14, 15]. The risk-of-bias tool recommended by the Cochrane Handbook [16, 17] was used for evaluating of risk of bias in each included study. The components for risk of bias evaluation included (1) selection bias; (2) group hidden; (3) blinding method of both doctors and patients; (4) result evaluation blind method; (5) completeness of the report results; (6) reporting bias; and (7) other biases. In this paper, if the score meets the index, it is the low risk. But, if it does not, it is the high risk. And if the score is unclear, it is the unclear risk.

The article "Exercise Intervention Improves Blood Glucose Levels and Adverse Pregnancy Outcomes in GDM Patients: A Meta-Analysis" was published in 2022. Journal: Comput Math Methods Med.

### 2.4. Statistical Analysis

The Review Manager (RevMan) 5.3 software was used for statistical analysis. For continuous variables, fasting blood glucose, 2-h postprandial blood glucose and glycosylated hemoglobin (HbA1C), and mean difference (MD) with 95% CI were pooled. For dichotomous variables such as preterm birth rate, cesarean section rate, neonatal macromorbidity rate, premature rupture of membranes rate, and neonatal hypoglycemia rate, relative risk (RR) and 95% CI were used as effect indicators. The *I*^2^ and *P* tests were carried out for assessing interstudy heterogeneity. In the presence of *P* < 0.10 and *I*^2^*≤ 50%*, the fixed-effect model was used. Otherwise, the random-effect model was used. A two-sided *P* < 0.05 was regarded to denote statistical significance.

## 3. Results

### 3.1. Literature Screening Results

A total of 1420 studies were retrieved from the database, including 1168 English publications and 252 Chinese publications. After removing duplicate publications, 935 literature remained. By browsing the title and abstract of the literature, 925 studies were excluded. Finally, 9 English literature were included in this study for analysis (Figure 1), including 4 high-quality literature and 5 medium-quality literature. The risk-of-bias assessment of each included publication is shown in Figure 2.

### 3.2. Overall Characteristics of Included Literature

Data from a total of 1289 GDM patients from 9 studies were meta-analyzed. Four papers used mild-intensity exercises such as strolling, brisk walking, cycling, and stretching, and 5 papers used moderate-intensity exercises such as resistance, aerobic, gymnastics, and yoga. The exercise time ranged from 30 to 60 minutes. The main outcome indicators were fasting blood glucose, 2-h postprandial blood glucose, premature birth, cesarean section, and neonatal macrosomia. The secondary outcome indicators were HbA1c, premature rupture of membranes, and neonatal hypoglycemia. Detailed information for the 9 included studies are listed in Table 1.

The article "Exercise Intervention Improves Blood Glucose Levels and Adverse Pregnancy Outcomes in GDM Patients: A Meta-Analysis" was published in 2022. Journal: Comput Math Methods Med.

### 3.3. Meta-Analysis Results

#### 3.3.1. Effect of Exercise on Fasting Blood Glucose in Patients with GDM

A total of 9 studies [2, 3, 9–14] with 1289 subjects, including 647 in the interventional group and 642 in the control group, reported the effect of exercise on fasting blood glucose in GDM patients. The heterogeneity test was performed on the included subjects (*I*^2^ = 96%, *P* < 0.00001), and the random effect model analysis was used, MD = −0.22, *95% CI* (-0.47, 0.03). Brisk walking, walking, and stretching/cycling were divided into mild exercise groups [*MD* = −0.35, 95% CI (-0.96, 0.26), *Z* = 1.13, *P* = 0.26], and the rest were moderate exercise groups [*MD* = −0.11, 95% CI is (-0.23, 0.01), *Z* = 1.75, *P* = 0.08] according to the type of exercise. Combined analysis of the two groups, MD was -0.22, 95% CI was (-0.47, 0.03), combined effect size test *Z* = 1.73, *P* = 0.08, indicating that different exercises in the two groups had no effect on fasting blood glucose in patients with GDM (Figure 3). Analysis between the two groups showed no significant difference (*P* = 0.44).

#### 3.3.2. Effect of Exercise on 2-h Postprandial Blood Glucose in Patients with GDM

Significant heterogeneity between studies was observed (*I*^2^ = 93%, *P* < 0.001). Random-effect model showed that exercise could significantly reduce 2-h postprandial blood glucose in GDM patients (MD = −0.62, *95% CI* (-0.91 to -0.34), *Z* = 4.29, *P* < 0.001, Figure 4).

#### 3.3.3. Effect of Exercise on HbA1c

In total, 4 studies [3, 9, 11, 14] that included 330 controls and 350 from the interventional group assessed the effect of exercise on HbA1c in patients with GDM. As shown in Figure 5, the meta-analysis performed with the random-effect model (*I*^2^ = 97%, *P* < 0.001) found that exercise could significantly reduce HbA1c in GDM patients (MD = −0.47, *95% CI* (-0.81 to -0.13), *Z* = 2.69, *P* = 0.007).

#### 3.3.4. Effect of Exercise on the Premature Birth Rate

There was no heterogeneity, for which the fixed-effect model analysis was used. Meta-analysis using data pooled from 7 studies [2, 3, 9–13] that included 1081 patients indicated that exercise did not affect preterm birth rate in GDM patients [pooled effect size *RR* = 0.78, 95% CI (0.46, 1.32), *Z* = 0.93, and *P* = 0.35, Figure 6].

#### 3.3.5. Effect of Exercise on Cesarean Section Rate

The effect of exercise on the cesarean section rate was reported in 8 studies [2, 3, 9–13] that included 562 cases in the interventional group and 557 in the control group. The cesarean section rates were 29.71% in the interventional group and 36.98% in the control group. The pooled analysis (Figure 7) using the fixed-effect model (*I*^2^ = 0%, *P* = 0.55) suggested that exercise could significantly reduce the rate of cesarean section rate (RR = 0.83, 95% CI 0.71-0.98, *Z* = 2.25, *P* = 0.02).

The article "Exercise Intervention Improves Blood Glucose Levels and Adverse Pregnancy Outcomes in GDM Patients: A Meta-Analysis" was published in 2022. Journal: Comput Math Methods Med.

#### 3.3.6. Effect of Exercise on the Incidence of Neonatal Macrosomia

Neonatal macrosomia born to GDM patients were assessed in 5 studies [2, 10–13] that included 381 patients in the interventional group and 392 in the control group. Macrosomia was noted in 21 cases (5.51%) in the interventional group and 38 in the control group (9.69%). As outlined in Figure 8, the combined effect calculated using the fixed-effect model (*I*^2^ = 0%, *P* = 0.48) shows an RR of 0.57 (*95% CI* 0.34-0.95, *Z* = 2.17, *P* = 0.03), indicating that exercise could significantly reduce the risk of giving birth to newborns with macrosomia in GDM patients.

#### 3.3.7. Effect of Exercise on the Incidence of Premature Rupture of Membranes

The RR pooled from 4 publications that included 227 patients in the interventional group and 281 patients in the control group was 0.84 (*95% CI* 0.53-1.34, *Z* = 0.72, *P* = 0.47) from the fixed-effect model (*I*^2^ = 0%, *P* = 0.56) and suggested that exercise did not significantly reduce the incidence of premature rupture of membranes (Figure 9).

#### 3.3.8. Effect of Exercise on the Incidence of Neonatal Hypoglycemia

Data combined from a total of 388patients, including 190 in the interventional group and 198 in the control group with the fixed-effect model (*I*^2^ = 0%, *P* = 0.83), showed that exercise did not significantly reduce the risk of neonatal hypoglycemia (RR = 0.31, *95% CI* 0.09, 1.10, *Z* = 1.81, *P* = 0.07, Figure 10).

## 4. Discussion

In this study, we pooled data from 9 RCTs, including 4 high-quality and 5 medium-quality studies. The risk-of-bias assessment indicated that 4 publications were of low risk, and the other 5 were at medium risk for bias. A total of 1289 pregnant women diagnosed with GDM were included. The results showed that exercise during pregnancy had a positive effect GDM by significantly improving blood glucose control, such as fasting blood glucose, 2-h postprandial blood glucose, and HbA1c. This finding was consistent with the results of other studies [7, 18, 19]. In this meta-analysis, the forest maps showed that the pooled MD for fasting blood glucose, 2-h postprandial blood glucose, and HbA1c were -0.22, -0.62, and -0.47, respectively, indicating that mild to moderate physical exercise could effectively manage blood glucose level in GDM. This result was consistent with the recommendations of some guidelines [7, 20], and exercise could improve blood glucose control in the state of insulin resistance [21]. Therefore, exercise for about 150 minutes a week could reduce the blood glucose level of people with impaired glucose tolerance. Some previous studies have shown that this exercise can also reduce the risk of future type 2 diabetes mellitus in GDM patients [13], among which resistance exercise was better, and aerobic exercise had the best effect [22, 23].

The article "Exercise Intervention Improves Blood Glucose Levels and Adverse Pregnancy Outcomes in GDM Patients: A Meta-Analysis" was published in 2022. Journal: Comput Math Methods Med.

Premature birth and macrosomia neonatorum are common adverse pregnancy outcomes [3, 10, 24]. Previous studies reported that these adverse outcomes were closely related to overweight and GDM [12, 22, 25]. Hence, it is particularly important to take certain interventions during pregnancy to prevent the incidence of premature and macrosomia [26, 27]. The meta-analysis results in this study showed that exercise intervention could reduce the incidence of premature infants and macrosomia. The cesarean section rate in the exercise intervention group was 29.71%, which was significantly lower than that in the control group. The incidence of macrosomia in the exercise intervention group was 5.51%, which was also lower than that in the control group. However, the incidence of other adverse outcome indicators, such as premature delivery, premature rupture of membranes, and neonatal hypoglycemia, did not differ significantly between the exercise group and control group.

This study showed that exercise intervention could improve the blood glucose level of GDM patients (fasting blood glucose, 2-h postprandial blood glucose, and HbA1c) and reduce adverse pregnancy outcomes (premature birth and macrosomia), which was consistent with some research results. Therefore, exercise has an excellent therapeutic effect on the treatment of GDM and could reduce the incidence of adverse pregnancy outcome for GDM patients. However, this study also had some shortcomings. For example, we only searched the commonly used databases, which might have omitted other potential publications. In addition, only 9 literature that met the inclusion/exclusion criteria were included. Some indicators of these articles were not clearly defined. And these literature come from different countries and regions, and the original exercise habits may be different. At last, not all exercise methods with the same intensity and frequency were used in exercise activities, which might introduce potential sources for inter-study heterogeneity. The differences in the age of the patients enrolled in this paper and the differences in exercise activities that do not all use the same way, intensity, and frequency of exercise methods will lead to certain limitations in this paper.

## 5. Conclusion

1. Exercise intervention improves the blood glucose level of GDM patients, such as 2-h postprandial blood glucose and HbA1c
2. Exercise intervention reduces adverse pregnancy outcomes, such as premature birth and macrosomia

The article "Exercise Intervention Improves Blood Glucose Levels and Adverse Pregnancy Outcomes in GDM Patients: A Meta-Analysis" was published in 2022. Journal: Comput Math Methods Med.

## Figures and Tables

**Figure 1:** Flow chart of included literature screening.

**Figure 2:** Risk-of-bias assessment of each included literature.

**Figure 3:** Forest diagram of the effect of exercise on fasting blood glucose in patients with GDM.

**Figure 4:** Forest diagram of the effect of exercise on 2-h postprandial blood glucose in patients with GDM.

**Figure 5:** Forest diagram of the effect of exercise on glycosylated hemoglobin (HbA1c) in patients with GDM.

**Figure 6:** Forest diagram of the effect of exercise on the premature birth rate of GDM patients.

**Figure 7:** Effect of exercise on cesarean section rate of GDM patients.

**Figure 8:** Effect of exercise on the incidence of neonatal macrosomia in patients with GDM.

**Figure 9:** Forest diagram of the effect of exercise on the incidence of premature rupture of membranes in GDM patients.

**Figure 10:** Forest diagram of the effect of exercise on the incidence of neonatal hypoglycemia in GDM patients.

**Table 1:** General information of the literature included in this study.

Included literature	Country	Study type	Sample size		Exercise interventions			Exercise time (min)	Outcome indicators
			Experimental group	Control group	Movement mode	Frequency	Intensity		
Bo [13]	Italy	RCT	101	99	Brisk walking	Daily	Mild	20	①②④⑤⑥⑦
Chen [8]	China	RCT	79	60	Strolling	Daily	Mild	30	①②③④⑤
Ding [14]	China	RCT	210	218	Strolling	Daily	Mild	60	①②④⑤⑥⑧
Guelfi [11]	Australia	RCT	85	84	Stretch/ride	2-3 times a week	Mild	60	①②③④⑤
Jin [12]	China	RCT	65	66	Gymnastics	3 times a week	Moderate	50	①②④⑤⑥⑦⑧
Kokic [4]	Australia	RCT	18	20	Aerobic/resistance exercise	3 times a week	Moderate	50-55	①②⑤⑥
Sununta [15]	Thailand	RCT	85	85	Yoga	3 times a week	Moderate	45	①②③
Wu [2]	China	RCT	75	75	Aerobic/resistance exercise	5 times a week	Moderate	30	①②④⑤⑥
Zhao [3]	China	RCT	43	46	Resistance exercise	3 times a week	Moderate	50-60	①②④⑤⑥⑦⑧

Note: ① Fasting blood glucose; ② blood glucose 2 hours after a meal; ③ glycosylated hemoglobin (HbA1c); ④ premature birth; ⑤ cesarean section; ⑥ neonatal macrosomia; ⑦ premature rupture of membranes; ⑧ neonatal hypoglycemia.

## Data Availability

The data used and analyzed during the current study are available from the corresponding author.
